RETRACTED

# Serum Exosomal MicroRNAs Predict Acute Respiratory Distress Syndrome Events in Patients with Severe Community-Acquired Pneumonia

**DOI:** 10.1155/2019/3612020

**Published:** 2019-08-05

**Authors:** Xu Wu, Chengzhi Wu, Wenyu Gu, Haiying Ji, Lei Zhu

**Affiliations:** ^1^Department of Pulmonary Medicine, Zhongshan Hospital, Fudan University, Shanghai, 200032, China; ^2^Department of Laboratory, Qihe People's Hospital, Dezhou, 251100, China; ^3^Department of Urology, Shanghai Tenth People's Hospital, Tongji University School of Medicine, No. 301, Yanchang Rd., Shanghai, 200072, China

## Abstract

**Background:**

Severe community-acquired pneumonia (SCAP) requiring intensive care unit (ICU) treatment commonly causes acute respiratory distress syndrome (ARDS) with high mortality. This study was aimed at evaluating whether microRNAs (miRNAs) in circulating exosomes have the predictive values for patients at risk of developing ARDS due to SCAP.

**Methods:**

ARDS/ALI-relevant miRNAs were obtained by literature search. Exosomes in serum were isolated by ultracentrifugation method and identified by Transmission Electron Microscopy. Then the miR profiling in the exosomes using real-time PCR was analyzed in SCAP patients with or without ARDS. Moreover, multivariate Cox proportional regression analysis was performed to estimate the odds ratio of miRNA for the occurrence of ARDS and prognosis. The receiver operating characteristics (ROC) curves were calculated to discriminate ARDS cases. Finally, the Kaplan-Meier curve using log-rank method was performed to test the equality for survival distributions with different miRNA classifiers.

**Results:**

A total of 53 SCAP patients were finally recruited. Ten miRNAs were picked out. Further, a subset of exosomal miRNAs, including the miR-146a, miR-27a, miR-126, and miR-155 in ARDS group exhibited significantly elevated levels than those in non-ARDS group. The combined expression of miR-126, miR-27a, miR-146a, and miR-155 predicted ARDS with an area under the curve of 0.909 (95 % CI 0.815 –1). Only miR-126 was selected to have potential to predict the 28-day mortality (OR=1.002, P=0.024) with its median value classifier.

**Conclusions:**

The altered levels of circulating exosomal microRNAs may be useful biologic confirmation of ARDS in patients with SCAP.

## 1. Introduction

Acute respiratory distress syndrome (ARDS) is a life-threatening disease with a current mortality of about 40% [1]. Severe community-acquired pneumonia (SCAP) is the most frequent cause of ARDS. Despite modifications on clinical definition [2], ARDS patients remain non-specific, not uniformly diagnosis with heterogeneous etiologies or complexity of pathologies, thus responding differently to therapeutic interventions [3]. Therefore, identification of potential biomarkers that facilitate diagnosis of ARDS could improve clinical care and could be used to enroll a more homogeneous group of patients into clinical practice with effective therapies.

RETRACTED

It is unlikely that a single biomarker will have adequate specificity for the clinical confirmation of ARDS in patients who have developed pneumonia. MicroRNAs (miRNAs) play crucial roles in the posttranscriptional regulation of gene expression in pathogenesis of lung diseases and infections [4]. Circulating exosomes are membrane vesicles shed by a variety of blood or endothelial cells, and have been shown to be important mediators of intercellular communication and microenvironment, holding the potential to miRNAs delivery [5]. In the presence of devastating stimuli, the compositions of exosomes including miRNAs, could be robustly altered, thus accumulating studies center round the potentials of exosomes to serve as promising biomarkers [6, 7]. Currently, the content of circulating exosomes in patients with or without ARDS remains elusive. As miRNAs have to be used to construct prognostic classifier for early prediction of disease outcomes [8], it is not yet clear if the biological significance of exosomal miRNAs is superior to a combination of abnormal biomarkers. Although the definition of ARDS is based on clinical criteria, no studies have tested the possible value of a panel of exosomal miRNAs to assist in the diagnosis of ARDS in patients with SCAP.

Therefore, our purpose is to confirm whether the exosomal miRNAs could be used as biomarkers for discriminating the patients at risk of developing ARDS due to SCAP. Herein, we tentatively filtrated a group of ARDS/ALI-relevant miRNAs through several literatures. Then, these profiles of miRNAs carried by exosomes in serum were examined. We also evaluated the association of aberrant exosomal miRNAs expressions with the clinical pathological properties and prognosis, which is probably helpful for understanding of pathogenesis and accurate diagnosis in SCAP patients.

## 2. Methods

### 2.1. Subject Recruitment and Sample Acquisition

This prospective, observational study was conducted in the intensive care unit (ICU) of Zhongshan hospital. The consecutive patients suspected of CAP were enrolled from November 2016 to May 2018. CAP was defined as the presence of a new infiltrate on a chest radiograph and at least one of the following signs and symptoms: cough, sputum production, dyspnea, core body temperature > 38.0°C, auscultatory findings of abnormal breath sounds, and rales according to the American Thoracic Society (ATS) criteria, and its severity was evaluated by pneumonia severity index (PSI). Exclusion criteria included pregnancy, terminal illness (malignant cancer of any type, end-stage liver, or renal disease), severe immunosuppression, and refusal of informed consent. Additional exclusion criteria were, prior hospitalization within 15 days before admission, pneumonia developing during hospitalization, and delayed ICU admission for more than 48 hours. The study was approved by the Ethics Committee of the Fudan University (Approval number B2017-061R) and conducted with informed consent forms obtained from all participants.

RETRACTED

Demographic information from severe CAP patients was collected including baseline clinical variables, blood PO_2_/FiO_2_ ratio, laboratory data as well as outcome. The daily clinical variables of interest were recorded to calculate the Acute Physiology and Chronic Health Evaluation II (APACHE II) scores and sequential organ failure assessment (SOFA) scores [9]. During the patient's hospital stay, we evaluated the presence of ARDS that defined by the Berlin definition [2]. Co-morbidities during hospitalization, style of invasive ventilator parameters and hospital stay days were documented for each patient. Also, a follow-up at 28-day mortality was performed to evaluate the prognosis. After enrollment of patients, data was blinded to avoid potential bias.

Blood samples from consenting subjects were collected within 24 hours of admission to the ICU. All biomarkers were assayed in duplicate in thawed serum at enrollment using commercially available ELISAs (IL-6, IL-10, vWF and ANG2, R&D Systems).

Biomarker concentrations were measured on a Bio-Plex System 100 (Bio-Rad, Hercules, CA, USA). Additionally, serum was separated via centrifugation at 1,500 g for 15 min at 4°C, followed by a second centrifugation at 16,000 g for 10 min at 4°C to eliminate residual cells debris. In order to prevent exosomes degradation and loss, samples should be handled within 30 minutes after blood withdrawal.

### 2.2. Candidate miRNA Selection

Using the combination of keywords and MeSH terms for “ALI” and “microRNA”, we searched PubMed for articles that describe associations between the miRNAs and ARDS. To focus on the miRNAs with a high likelihood of relevance, we considered only miRNAs with at least two published references to be potential candidates for investigation. These cross-referenced with miRNA expression data were performed on serum-derived exosomes.

### 2.3. Bioinformatic Analysis

The databases TargetScan and miRanda were performed to identify experimentally validated and predicted gene targets of differentially expressed exosomal microRNAs.

RETRACTED

Subsequently, these genes were input into DAVID Database (http://david.abcc.ncifcrf.gov/) and the Kyoto Encyclopedia of Genes and Genomes (KEGG) for Gene Ontology (GO) or pathway enrichment analysis. The enrichment of related genes in three major GO classifications, that is, cell components (CC), biological processes (BP), and molecular functions (MF). KEGG pathway analysis was carried out to analyze the canonical pathways of relevance to ALI/ARDS. A network graph for these exosomal miRNAs was generated via the cytoscape software, directly showing the association of these genes with miRNAs.

### 2.4. Serum Exosomes Isolation from Serum and Identification

The size and morphology feature of exosomes were examined by Transmission Electron Microscopy (TEM). Firstly, prepared serum was ultra-centrifuged at 100,000 x g for 120 minutes. Following ultracentrifugation, the supernatant was aspirated and the exosome pellets were re-suspended in 50 ul PBS. For visualization of samples using TEM, exosome suspensions were prepared on formvar-coated copper-palladium grids and negatively stained with uranyl acetate. Image acquisition was conducted using a JEOL 1200EX TEMSCAN electron microscope at Fudan University. The remaining pellets containing the exosome fractions were diluted in sterile PBS for cell treatment or stored up to 6 months for PCR analysis at -80°C. For exosomal total RNA, the pellet fractions were washed twice with PBS and lysed with Trizol. Total RNA was quantified by the NanoDrop ND-2000 (Thermo Scientific) and the RNA integrity was assessed using Agilent Bioanalyzer 2100 (Agilent Technologies).

### 2.5. Quantitative Validation of miRNAs by Real-Time PCR

Total exosomal RNAs extracted from 250 *μ*l serum were polyadenylated and reverse-transcribed with a poly (T) adapter into cDNAs. The reverse transcription reaction was carried out with PrimeScript™ II reverse transcriptase (Takara, Japan) at 42°C for 60 min, and 75°C for 15 min in a total volume of 10 *μ*L. To measure the candidated miRNA levels, fold changes were tested by quantitative PCR amplification with SYBR PrimeScript miRNA RT-qPCR Kit (Takara, Japan). All reactions were run in triplicate. Specificity of the RT-qPCR product was confirmed with melting curve analysis. Ct values were determined using default threshold setting. miRNAs with a Ct value of more than 40 and a detection rate of less than 75% in any group were excluded from further analyses. Moreover, miR-39 was used as an endogenous control. Relative fold change of miR expression normalized to miR-39 was calculated using the 2^-ΔΔCt^ method.

### 2.6. Statistical Analysis

Results for normally distributed continuous variables are presented as mean ± standard deviation and compared between groups by Student's* t* tests (paired groups) or Mann–Whitney U test (unpaired groups). Results for categorical variables are presented as sample rate (constituent ratio) and were compared Chi-squared test. Binary logistic regression analysis was carried out to determine the independent predictors of the occurrence of ARDS or the 28-day mortality. The discriminatory power of each scoring index was measured by receiver operating characteristic (ROC) curves. The areas under the ROC curve (AUC) was calculated to give an estimate of the overall accuracy of each scoring index in predicting different patient outcomes (occurrence of ARDS and 28-day mortality). An area of 0.50 implies that the scoring index is no better than chance, whereas an area of 1 implies perfect accuracy. Spearman correlation analysis was applied to determine the correlation between miRNAs, vWF, ang-2, IL-6, IL-10 and SOFA or APACHE II score. The Kaplan–Meier (KM) curve was generated to evaluate the association between the levels of miR-126/146a and survival rate with log-rank test. All tests were two-sided and the statistical significance was assumed at a value of P<0.05.

RETRACTED

## 3. Results

### 3.1. Characteristics of Enrolled Subjects

A total of 68 patients suggestive of severe CAP were admitted during the study enrollment period. Of the 59 patients who signed consent forms, 6 were excluded because of inadequate laboratory data. Ultimately, 53 were included in the study. The general demographic data, co-morbidities, and associated laboratory findings of enrolled subjects were detailed in Table 1. There were no significant differences between ARDS and non-ARDS groups with respect to sex, age and medical history. In contrast, oxygenation index (PO_2_/FiO_2_) in patients experiencing ARDS was lower than non-ARDS patients. Subjects who experienced SCAP had no significant differences in their rates of mechanical ventilation, as well as hospital lengths of stay. 28-day mortality rate increased in parallel with a rise in PSI, which tended to be higher in patients with ARDS. However, regarding to the APACHE II score, SOFA score, CRP, PCT, co-morbidities, and noninvasive ventilation parameters PEEP, no statistical differences were observed between them (P > 0.05).

### 3.2. The Altered Levels of Exosomal MicroRNAs in Patients with Severe Community-Acquired Pneumonia

Exosomes were purified from serum of SCAP patients using ultracentrifuge method and examined by electron microscopy. The electron micrographs of these revealed rounded structures with a size of approximately 25–75 nm (Figure 1). Meanwhile, these results confirmed the efficacy of our protocol for exosomes isolation.

RETRACTED

We identified 27 miRNAs associated with ARDS/ALI, and excluded those not measured or in very low levels. The remaining 10 miRNA were picked out and further analyzed, including miR-15a, miR-16, miR-26, miR-21, miR-27a, miR-181b, miR-126, miR-146a, miR-155, and miR-223. To comprehend the functions and potential mechanisms of exosomal miRNAs involved in ARDS pathogenesis, as a first approach, we identified these experimentally validated and predicted gene targets of miRNAs using TargetScan and miRanda databases. Further, the generated network via the cytoscape software was visualized as Figure 2. In addition, we put these genes input into the David Database for GO enrichment analysis, revealing 27 GO terms with statistical significance (P <0.05), shown as Figure 3. KEGG pathway showed seven potential pathways that miRNAs and their related genes got involved in ARDS.

Based on the presence or absence of ARDS, the mean expression levels of the candidate miRNA in serum-derived exosomes was determined by RT-PCR and displayed in Figure 4. The levels of serum exosomal miR-146a, miR-27a, miR-126, and miR-155 were significantly higher in patients with ARDS than in those without (P = 0.004, P = 0.005, P = 0.008, P = 0.014, respectively). Meanwhile, the levels of miR-223 and miR-181b were significantly lower in patients with ARDS than in those without (P = 0.001 and P = 0.038). As PSI, PO_2_/FiO_2_ and some miRNAs levels were significant different between ARDS and non-ARDS groups, a Pearson linear correlation matrix analysis was further performed. Upregulation of miR-126 was correlated with the severity of ALI as reflected by PSI (r= 0.397, P=0.036). The inverse association between pronounced miR-126 levels and PO_2_/FiO_2_ was, however, not so significantly evident (r= -0.033, P=0.814). Additionally, miR-16 was inversely related to the PO_2_/FiO_2_ (r= -0.369, P=0.007). We found significant positive correlation between miR-146a and APACHE II score (r= 0.323, P=0.018), while no associations existed between other miRNA levels and APACHE II score. Furthermore, our study shows that SOFA score did not relate to any exosomal miRNAs. Patients with higher SOFA scores, regardless of ARDS occurrence, did not have a significant trend toward higher mortality rate at enrollment. An overview graph of the above significant linear correlations is given in Figure 5.

With regard to the biomarkers in various aspects of the pathophysiology of ARDS, biomarker panel that includes biomarkers of pulmonary endothelial injury or inflammation may be the most useful for discriminating the patients with ARDS. It is hypothesized that circulating angiopoietin-2 and vWF were generated by the lung endothelium, and associated with pulmonary severity of ALI. To further study clinical significance, we evaluated whether IL-6, Ang-2, IL-10 and VWF levels correlated with the development and clinical outcomes of ARDS. As expected, higher vWF concentrations were significantly found in patients classified in occurrence of ARDS group. Decreased IL-10 levels in parallel with a rise in IL-6 were also assessed among the two patient categories. In all, a Spearman analysis for the correlation coefficients of differentially expressed exosomal miRNAs with IL-6, Ang-2, IL-10, and vWF levels is demonstrated in Table 2.

RETRACTED

### 3.3. The Predictive Value of Differentially Expressed Exosomal miRNAs for ARDS Events

All factors affecting the occurrence of ARDS in SCAP patients were analyzed in multivariate Cox proportional logistic regression. The area under the curve (AUC) values for individual miRNAs ranged between 0.592 and 0.779 as presented in Table 3. Exosomal miR-126 was the most predictive single miRNA for distinguishing SCAP patients with or without ARDS with an AUC of 0.779 [95 % confidence interval (CI) 0.652-0.906]. In a logistic regression model, after adjusting for other confounding factors such as age, sex, co-morbidities, and associated laboratory, miR-126 were independent predictors in SCAP patients for the risks of ARDS (OR = 1.013, P < 0.001). As a predictor variable, miR-27a was also independently associated with the presence of ARDS (OR = 1.01, P = 0.001). Indeed, multivariate logistic regression analysis with occurrence of ARDS as an outcome showed that elevation of circulating exosomal miR-146a predicted ARDS (regression coefficient=1.071, P=0.014). A high correlation coefficient was observed in miR-155 in the development of ARDS (OR = 1.44, P = 0.015). The final multiple marker model included the combination of miR-126, -27a, -146a and -155. The receiver operating characteristics (ROC) curves for miR-126 and miR-146a and the multiple marker model were calculated to differentiate ARDS cases from non-ARDS controls as shown in Figure 6. Taken together, the AUC for the multiple marker model was larger than any individual marker [AUC = 0.909 (95% CI 0.815 – 1)]. The ROC curves for ARDS events showed that a combination of miR-126, -27a, -146a, and -155, in contrast to miRNAs alone, were of predictive value.

### 3.4. Changes in Exosomal MicroRNAs Reflect ARDS Progression

The final miRNA classifier was obtained by both most differential expression and backwards elimination. In a second set of analyses with 28-day mortality, exosomal miRNA with a potential prognostic role is miR-126, whose expression was obviously higher in non-survivors than those who survived (OR=1.002, P=0.024). To further evaluate the predictive accuracy, we also divided the patients into two groups according to median value. Expression of miR-126 classifier larger than median was assigned as high expression, lower than median was assigned as low expression. The Kaplan–Meier survival curves and log-rank test for 28-day mortality were illustrated in Figure 7. There is a clear tendency that SCAP patients with higher concentration of miR-126 had increased mortality. MiR-146a was also shown to have prognostic utility, but did not reach statistical significance (OR=0.71, P=0.064). However, using the miR-146a classifier, the Kaplan– Meier curve showed statistical difference on 28-day survival rate between the above cutoff group and the below cutoff group, when miR-146a levels were stratified by the cutoff 4.

RETRACTED

Of note, APACHE II score alone was not predictive for 28-day mortality in SCAP patients in receiver operating characteristic curves (minimum area under the curve=0.415, P=0.295). In addition, AUCs of miR-126, miR-155, miR-27a, miR-146a in combination with APACHE II scores were 0.698, 0.59, and 0.664, 0.682 for predicting 28-day mortality, respectively. Thus, these AUCs were lower than those of miRNAs alone (all P < 0.05).

## 4. Discussion

The introduction of exosome served as vehicles of miRNAs, has shed light on novel biomarker discovery. The major finding of the present study demonstrated that levels of some exosomal miRNAs were markedly different in patients with SCAP experiencing ARDS or not. In contrast, conventional indicators such as APACHE II, CRP and PCT showed no statistical difference. Modifications in expressive patterns of exosomal miRNAs could regulate the endothelial function, inflammatory response and tissue repair mechanisms, all of which contribute to endothelial activation and barrier injury in the setting of ALI/ARDS. In addition, four abnormal exosomal miRNAs in serum provided excellent discrimination for the diagnosis of ARDS as assessed by ROC curve analysis. Specific exosomal miRNAs also represented the potentially suitable biomarkers of SCAP progression. In particular, exosomal miR-126 is an independent predictor of ARDS events and 28-day mortality, reflecting the severity of SCAP. Therefore, exosomes offer innovative possibilities in detecting and monitoring the development of ARDS evoked by SCAP.

MicroRNA regulation of cellular processes is a complicated issue as each specific miRNA can have a multitude of mRNA targets. Our goal was to investigate possible cellular mechanisms influencing occurrence of ARDS in acute inflammatory response and endothelial injury associated with SCAP. Four of the pathways appeared to be particularly relevant to ARDS including LPS-stimulated MAP kinase signaling, mTOR and Jak-STAT signaling, and cell cycle signaling. The role of miRNAs in pulmonary disease are mostly based in animal models, thus the degree of translation into human medicine is unclear. Although few miRNAs have been detected in the pathogenesis of pneumonia, Abd-El-Fattah et al. demonstrated that miR-155 and miR-21 were markedly increased in patients with pneumonia [10]. Functional miRNAs are capsulated in exosomes and delivered to recipient cells, subsequently regulating gene expression by binding to targeted mRNAs to inhibit their translations. In our separate analysis, the decreased levels of exosomal miR-181b could be explained by the evidence that, it inhibits nuclear factor-*κ* -gene binding (NF-*κ*B)-mediated endothelial cell activation and vascular inflammation in response to the injury [11]. Wang et al. reported that miR-27a was up-regulated and promoted inflammatory response in sepsis, which was concordant with the elevated expression of exosomal miR-27a in our study [12]. It has been established that alterations in certain miRNAs during ARDS might participate in the modulation of the inflammatory process and tissue repair, as these changes are concomitant to the levels of the inflammatory mediators as well as the recruitment of immune cells in the lung [13, 14]. For example, miRNAs such as miR-146a and miR-155 play crucial roles in regulating the immune response by modulating components of NF-*κ*B signaling [15]. Li et al. demonstrated that miR-15a, miR-16 and miR-223 were found to target the IKK-*α* expression, and decreased expression of these miRNAs led to an increase in IKK-*α* in human monocytes [16]. Moreover, ectopic expression of miR-146a could affect IL-6 secretion in primary human fibroblast. Goodwin et al. reported that the down-regulation of exosomal miR-15a and miR-27a may help to reliably identify ICU patients who develop septic shock [17]. These findings were only in good accordance with Poon et al. who have also shown that increased plasma exosomal miR-223 expression during cardiac surgery might play homeostatic roles in downregulating inflammatory responses through intercellular communication [18]. In light of the recent evidence, it may be speculated that, the suppressive role of miR-15a/16 on inflammatory genes might be overruled by the miR-223 leading to an enhanced production of anti-inflammatory factors in ARDS group.

RETRACTED

Endothelial dysfunction is a key characteristic of ARDS, giving rise to increasing vascular permeability and then pulmonary edema induced respiratory failure [19]. Considering that miR-126 regulates vascular integrity and angiogenesis by enhancing the actions of VEGF [20], previous study revealed that miR-126 contained in endothelial cell-derived MPs promoted vascular regeneration [21, 22]. Additionally, a significant loss of miR-126 defining the impaired regenerative capacity was reduced in diabetic patients [23]. However, a single endothelial stress can cause microparticles shedding without any cell damage or apoptosis, displaying vector functions for the intercellular exchange of biological information [24]. It can be postulated that miR-126 is largely induced by inflammatory response, thus explaining the elevated miR-126 levels in presence of ARDS. As an endothelial cell-restricted miRNA, miR-126 has been shown to be abnormally expressed in septic patients and correlated with a decreased survival, supporting its possible use as targetable biomarker for early detection and prognosis of ARDS. In regard to miR-126, exosomes represent its major serum compartment, whereas other miRNAs are predominantly found to be transported in the vesicle-free form [25]. Furthermore, exosomes can protect the bioactive substances from repeated freezing and thawing, enzymatic digestion (RNase), degradation, and other adverse conditions. In particular, exosomal miRNAs are stable in the circulation [26].

Our data indicated that the prognostic value of might be different in the case. Exosomes are actively released from cells with different phenotypes including lymphocytes, neutrophils, platelets, endothelial cells, or endothelial progenitor cells in a very selective manner [27], and must be transferred to s recipient cells to repress their target mRNAs, thus exerting different functions that correlated with the clinical course of critical diseases [28]. Nevertheless, these characteristics create a challenge to determining the exact cellular source of circulating miRNA. The complexity of pneumonia underlines the increasing recognition as a systemic disease with repercussions on other organs, not limited to the lung [29]. Regardless of the numerous exosome resources, we found that a combination of four miRNA markers in serum (miR-27a, miR-126, miR-146a, and miR-155) alongside clinical scores had improved prognostic values. In this context, our present study suggested that multi-functional exosomes containing both immune cell- and tissue-specific miRNAs with combined diagnostic values showed a great promise in comparison with other biomarkers.

Several limitations still existed in the present study. Only a selected number of miRs, based on previously published data, were analyzed. SCAP patients were mainly enrolled from the critical care unit of the pulmonary department, and suffered from multiple diseases. Accordingly, the high mortality rate in this small cohort may not be representative of general population of CAP patients. Although classifier containing exosomal miRNAs discovered in this study offered a potentially valuable advantage, novel exosomal miRNA signatures are incompletely recognized and warranted to better predict the prognosis or 28-day mortality in the clinical practice.

RETRACTED

To date, no single biomarker has sufficient discriminating power to clearly indicate prognosis in the personalized assessment of the patients [30]. Despite the definition of ARDS based on clinical criteria, altered levels of plasma biomarkers may assist in the precise diagnosis with possible ARDS, as well as potentially selecting patients into clinical practice for the optimization and modulation of intensive care.

## Figures and Tables

**Figure 1:** Isolation and characterization of serum exosomes with the standard ultracentrifuge method. (a) A representative electron microscopic image of exosomes showed the characteristic spherical shape and the size (25–75 nm). Scale bar=100 nm. (b) Analysis of the size distribution of exosomes isolated from individual serum.

**Figure 2:** TargetScan and miRanda databases identify several experimentally validated or predicted gene targets of these selected miRNAs in the context of ALI. The interactions between miRNAs (center) and its ambient genes construct the generated network via the cytoscape software.

**Figure 3:** Gene ontology (GO) and KEGG pathway analysis of ARDS-related genes are performed on DAVID database. The function enrichment of related genes in three major GO classifications, that is, cell components (blue), biological processes (green), and molecular functions (red).

**Figure 4:** Serum exosomal microRNAs from SCAP patients with or without ARDS were measured by real-time quantitative PCR. The values of the relative gene expression for target microRNA were normalized to miR-39 and calculated using the 2^−ΔΔCT^ method. Box plots are displayed where the horizontal bar represents the median, the box represents the IQR and the whiskers represent the maximum and minimum values. Comparisons made by Mann–Whitney U test. The values are expressed as the mean ± SEM. miRNA: microRNA, IQR: interquartile range.

**Figure 5:** Correlation between miRNAs and the severity of SCAP.

**Figure 6:** Receiver operating characteristics (ROC) curve analysis of miR-126 and miR-146a and the combination of multiple marker model for predicting the ARDS events in SCAP patients. Three ROC analyses are shown. Predicted probability of ARDS was computed from a multivariable logistic regression model that included the top four miRNA biomarkers.

RETRACTED

**Figure 7:** Kaplan–Meier survival analysis and log-rank test were used to evaluate the predictive values of miR-126 and miR-146a grouped by their expression levels.

**Table 1:** Baseline characteristics and outcome parameters in SCAP patients with and without ARDS.

Variables	ARDS (n=24)	Non-ARDS (n=29)	*P* value
*Age (yrs)*	59.63 ± 15.86	62.47 ± 12.10	0.078
*Sex (*%* men)*	18 (76%)	19 (67%)	0.209
*APACHE II score*	16.08 ± 9.41	12.83 ± 9.01	0.205
*SOFA score*	5.67 ± 3.55	4.45 ± 3.34	0.208
*PSI *	97.79 ± 28.38	95.31 ± 21.39	0.031
*PaO*_*2*_ */FIO*_*2*_ * ratio*	170.26 ± 105.49	226.47 ± 88.86	0.04
*Co-morbidities*			
(i) Pulmonary embolism, n (%)	2 (8%)	4 (14%)	0.541
(ii) Hypertension, n (%)	10 (42%)	10 (34%)	0.6
(iii) Diabetes mellitus, n (%)	6 (25%)	6 (21%)	0.715
(iv) COPD, n (%)	3 (13%)	9 (31%)	0.113
(v) Cardiovascular/cerebrovascular diseases, n (%)	6 (25%)	6 (21%)	0.715
*Complication*			
(i) Sepsis	7 (29%)	7 (24%)	0.686
(ii) AKI	3 (13%)	4 (14%)	0.893
*Platelet count (×10* ^*9*^ */L)*	181.5 ± 77.61	197.9 ± 108.9	0.539
*28-day mortality*	12 (50%)	10 (34%)	0.262
*Microbiological species *			
(i) Streptococcus pneumoniae	6 (25%)	6 (21%)	0.715
(ii) Haemophilus influenzae	1 (4%)	2 (7%)	0.676
(iii) Legionella pneumophila	0 (0%)	1 (3%)	0.368
(iv) Mycoplasma pneumoniae	1 (4%)	4 (14%)	0.241
(v) Other	9 (39%)	6 (21%)	0.151
(vi) unknown	7 (29%)	5 (17%)	0.311
*Invasive mechanical ventilation, n (*%)	16 (67%)	13 (45%)	0.116
*PEEP (cmH*_*2*_ *O)*	7.04 ± 4.73	4.86 ± 0.833	0.092
*Hospital stay, days*	20.17 ± 8.25	16.41 ± 8.42	0.109
*Laboratory parameters*			
(i) CRP (mg/dl)	90.27 ± 72.15	75.3 ± 58.43	0.408
(ii) Procalcitonin	1.75 ± 4.29	1.55 ± 3.76	0.858
(iii) Ang2 (ng/ml)	7.55 ± 1.67	5.08 ± 0.65	0.149
(iv) IL-6 (pg/ml)	62.04 ± 13.39	13.61 ± 2.01	0.002
(v) IL-10 (pg/ml)	10.66 ± 1.04	26.1 ± 7.53	0.07
(vi) vWF (% of control)	449.64 ± 118.45	266.64 ± 18.24	0.001

Data were presented as n (%), mean ± standard deviation. P value <0.05 was considered as statistically significant.

APACHE II, Acute Physiology and Chronic Health Evaluation II score; CRP, C-reactive protein; PSI, pneumonia severity index; SOFA score, Sequential Organ Failure Assessment score; CRP, C-reactive protein; PSI, pneumonia severity index; PEEP, positive end-expiratory pressure; Ang-2, angiopoietin 2; vWF, von Willebrand factor.

**Table 2:** Spearman analysis for the correlation of differentially expressed exosomal miRNAs with IL-6, Ang-2, IL-10, and vWF levels in SCAP patients.

Variables	vWF	IL-6	IL-10	Ang-2
*miR-126*				
(i) coefficient	0.836	0.245	-0.309	-0.063
(ii) *P* value	0.001	0.077	0.024	0.656
*miR-27a*				
(i) coefficient	0.144	0.636	-0.119	0.447
(ii)* P* value	0.302	0.001	0.397	0.001
*miR-181b*				
(i) coefficient	-0.27	-0.109	0.333	0.226
(ii)* P* value	0.051	0.435	0.015	0.103
*miR-223*				
(i) coefficient	0.552	0.288	-0.403	-0.034
(ii) *P* value	0.001	0.036	0.003	0.81
*miR-146*				
(i) coefficient	0.237	0.644	0.001	0.359
(ii)* P* value	0.088	0.001	0.993	0.008
*miR-155*				
(i) coefficient	0.16	0.335	0.081	-0.122
(ii)* P* value	0.252	0.014	0.565	0.383
*SOFA score*				
(i) coefficient	0.261	0.19	-0.199	-0.046
(ii)* P* value	0.059	0.173	0.154	0.741
*APACHE II score*				
(i) coefficient	0.092	0.098	-0.037	-0.019
(ii) *P* value	0.513	0.487	0.795	0.89

P value <0.05 was considered as statistically significant.

RETRACTED

Ang-2, angiopoietin 2; VWF, von Willebrand factor; APACHE II, Acute Physiology and Chronic Health Evaluation II score; SOFA score, Sequential Organ Failure Assessment score.

**Table 3:** Area under the curve (AUC) for individual miRNAs and for a multivariable logistic regression model.

Markers	AUC	95% CI	*P* value
miR-126	0.779	0.652-0.906	0.001
miR-27a	0.604	0.497-0.831	0.042
miR-146a	0.691	0.512-0.87	0.017
miR-155	0.592	0.429-0.755	0.253
miR-126+miR-27a	0.855	0.741-0.969	0.001
miR-126+miR-27a+miR-146a	0.876	0.761-0.991	0.001
miR-126+miR-27a+miR-146a+miR-155	0.909	0.815-1.00	0.001

miRNA: microRNA; CI: confidence interval.

P value <0.05 was considered as statistically significant.

## Data Availability

The data used to support the findings of this study are included in the article.

## Supplementary Materials

Supplementary Materials The raw experimental data of clinical parameters, serum exosomal microRNAs, and cytokines levels are provided as Supplementary Material 1.
